The article "Establishment and Verification of Logistic Regression Model for Qualitative Diagnosis of Ovarian Cancer Based on MRI and Ultrasound Signs" was retracted in 2023. Reasons: signs of a paper mill; compromised peer review; unreliable results or conclusions.

# Establishment and Verification of Logistic Regression Model for Qualitative Diagnosis of Ovarian Cancer Based on MRI and Ultrasound Signs

**DOI:** 10.1155/2022/7531371

**Published:** 2022-02-15

**Authors:** Xiao Guo, Guangcai Zhao

**Affiliations:** ^1^Department of Ultrasound, Qilu Hospital (Qingdao), Cheeloo College of Medicine, Shandong University, 758 Hefei Road, Qingdao, Shandong 266035, China; ^2^Department of Obstetrics and Gynecology, Qilu Hospital (Qingdao), Cheeloo College of Medicine, Shandong University, 758 Hefei Road, Qingdao, Shandong 266035, China

## Abstract

**Objective:**

To explore the establishment and verification of logistic regression model for qualitative diagnosis of ovarian cancer based on MRI and ultrasonic signs.

**Method:**

207 patients with ovarian tumors in our hospital from April 2018 to April 2021 were selected, of which 138 were used as the training group for model creation and 69 as the validation group for model evaluation. The differences of MRI and ultrasound signs in patients with ovarian cancer and benign ovarian tumor in the training group were analyzed. The risk factors were screened by multifactor unconditional logistic regression analysis, and the regression equation was established. The self-verification was carried out by subject working characteristics (ROC), and the external verification was carried out by K-fold cross verification.

**Result:**

There was no significant difference in age, body mass index, menstruation, dysmenorrhea, times of pregnancy, cumulative menstrual years, and marital status between the two groups (*P* > 0.05). After logistic regression analysis, the diagnostic model of ovarian cancer was established: logit (*P*) = −1.153 + [MRI signs : morphology × 1.459 + boundary × 1.549 + reinforcement × 1.492 + tumor components × 1.553] + [ultrasonic signs : morphology × 1.594 + mainly real × 1.417 + separated form × 1.294 + large nipple × 1.271 + blood supply × 1.364]; self-verification: AUC of the model is 0.883, diagnostic sensitivity is 93.94%, and specificity is 80.95%; K-fold cross validation: the training accuracy was 0.904 ± 0.009 and the prediction accuracy was 0.881 ± 0.049.

**Conclusion:**

Irregular shape, unclear boundary, obvious enhancement in MRI signs, cystic or solid tumor components and irregular shape, solid-dominated shape, thick septate shape, large nipple, and abundant blood supply in ultrasound signs are independent risk factors for ovarian cancer. After verification, the diagnostic model has good accuracy and stability, which provides basis for clinical decision-making.

## 1. Introduction

Ovarian cancer is the second malignant tumor of female reproductive system, with high malignant degree and rapid growth. Most patients have metastasized at the time of diagnosis, and the survival status is not optimistic. Its mortality rate is the highest among all malignant tumors of the female reproductive system [1, 2]. It is reported that with the growth of tumor, the five-year survival rate of patients with ovarian cancer gradually decreases, reaching 93% in stage I, 70%, 37%, and 25% in stage II, III, and IV, respectively [3]. In addition to malignant tumors, ovarian tumors also include many benign tumors, and the surgical resection effect is ideal [4]. At present, imaging examination is still the main examination method of ovarian tumors. Ultrasound diagnosis of ovarian tumors has the advantages of painless, simple operation and high repeatability and is widely used [5, 6]. Magnetic resonance imaging (MRI) has high resolution and spatial resolution for soft tissue, and it is widely used in the examination of abdominal and pelvic organ diseases, especially for the examination of ovarian tissue diseases [7, 8]. At present, MRI tends to be the best imaging choice for the diagnosis of ovarian cancer [9]. In this study, the logistic regression model of ovarian cancer diagnosis was established based on MRI and ultrasonic signs, in order to help clinical diagnosis and treatment effectively. The report is as follows.

The article "Establishment and Verification of Logistic Regression Model for Qualitative Diagnosis of Ovarian Cancer Based on MRI and Ultrasound Signs" was retracted in 2023. Reasons: signs of a paper mill; compromised peer review; unreliable results or conclusions.

## 2. Materials and Methods

A total of 207 ovarian tumor patients in our hospital from April 2018 to April 2021 were selected, of which 138 were used as the model creation training group and 69 were used as the model evaluation verification group. Patients enrolled from April 2018 to October 2020 are included in the model creation training group. Patients enrolled from November 2020 to April 2021 are included in the model evaluation verification group. We divide the training group into ovarian cancer group and benign ovarian tumor group according to whether the tumor of ovarian cancer patients is benign. Inclusion criteria: definite pathological diagnosis after operation; MRI and ultrasound were performed and the data were complete. The images could be used for diagnostic analysis; patient informed consent. Exclusion criteria: incomplete ultrasound, MRI, or pathological data; combined with severe organic diseases, such as coagulation dysfunction, renal insufficiency, heart failure, and other surgical contraindications; history of ovarian surgery; combined with other pelvic diseases, such as endometrial cancer and rectal cancer.

### 2.1. Methods

(1) Ultrasonography: Philips iu22, Philips IU elite, GE gyc2019-0068 color Doppler ultrasound diagnostic system, abdominal probe c5-1 (1 ~ 5 MHz), c1-5-d (1 ~ 6 MHz), vaginal probe c10-3v (3 ~ 10 MHz), and ic5-9-d (3 ~ 10 MHz). When the bladder is full, take the supine position for abdominal exploration, empty the bladder, and take the lithotomy position for vaginal ultrasonography. Two senior imaging doctors (with more than 5 years of experience) operated and analyzed the sonograms to observe the tumor location, shape, size, separation thickness, number of nipples, blood supply, nipple size, etc. When they disagree, they reached a consensus through consultation. All solid components ≥50% of the lesions are defined as solid, nipple height ≥7 mm is defined as large nipple, separation thickness ≥3 mm is defined as thick, and irregularity refers to one of the nonsmooth cystic wall, solid components, and nipples. Blood flow score: 1 point for no blood flow, 2 points for a small amount of blood flow, 3 points for moderate blood flow, 4 points for rich blood flow, and 3 and 4 points are defined as rich blood flow signals. (2) MRI examination: PHILIPS Ingenia 3.0 T magnetic resonance machine, scanning range: anterior superior iliac ridge to pubic symphysis level. Pelvic plain scan was performed on axial T1WI (TE and TR were 20 ms and 500 ms, respectively), axial T2WI (TE and TR were 100 ms and 4884 ms, respectively), axial T2WI-SPAIR (TE and TR were 65 ms and 2783 ms, respectively) and axial DWI-2B (TE and TR were 84 ms and 3000 ms, respectively, and TR is 80 ms and 2873 ms) and sagittal T2WI-SPAIR (TE and TR are 65 ms and 2752 ms). The horizontal slice thickness and interval are 5 mm and 1 mm, respectively, and the coronal slice thickness and interval are 5 mm and 1 mm, respectively. Gd-DTPA (0.4 mmol/kg and 2.0 ml/s) was injected, and the pelvic transverse arteriovenous scanning, pelvic sagittal scanning, and coronal delayed scanning were performed. With DYN mDIXON scanning, TE and TR were 1.32 ms and 3.7 ms, respectively, with a layer thickness of 3 mm and a layer distance of -1.5 mm. The images were independently read by two senior imaging doctors (with more than 5 years of experience). In case of disagreement, consensus was reached. When necessary, a third doctor with the same qualifications will participate in the judgment of the imaging results.

The article "Establishment and Verification of Logistic Regression Model for Qualitative Diagnosis of Ovarian Cancer Based on MRI and Ultrasound Signs" was retracted in 2023. Reasons: signs of a paper mill; compromised peer review; unreliable results or conclusions.

### 2.2. Observation Indicators

The observation indicators are as follows: (1) baseline data of patients, including age, body mass index, menstruation, dysmenorrhea, times of pregnancy, cumulative menstrual years, marital status, and tumor nature; (2) age, body mass index, menstruation, dysmenorrhea, times of pregnancy, cumulative menstrual years, marital status, MRI signs (shape, boundary, enhancement, and tumor components), and ultrasound signs (shape, solid, separated shape, big nipple, and blood supply) between patients with ovarian cancer and benign ovarian tumors; (3) multivariate analysis of influencing factors of ovarian cancer; (4) establishment and analysis of logistic regression model for ovarian cancer diagnosis; and (5) logistic regression model verification.

### 2.3. Statistical Treatment

The statistical software SPSS22.0 was used to process the data, and Bartlett variance homogeneity test and Shapiro-Wilk normality test were used to measure the data, all of which were confirmed to have variance homogeneity and approximately obey the normal distribution, described by ($\bar{x}\pm \text{s}$), and the independent sample *T*-test was used for comparison between groups. The data are expressed by *n* (%) and tested by *χ*2; the logistic regression was used to analyze the influencing factors of ovarian cancer, and a regression equation was established. The model's self-verification was evaluated by the area under the cure (AUC) of the receiver operating characteristic curve (ROC), and the K-fold cross validation was used for out-of-group verification, with *K* = 10. Two-sided test was used, *α* = 0.05.

## 3. Result

### 3.1. Clinical Baseline Data of the Patients

There was no significant difference in age, body mass index, menstruation, dysmenorrhea, times of pregnancy, cumulative menstrual years, marital status, and tumor nature between the two groups (*P* > 0.05). See Table 1.

### 3.2. Clinical Data of Patients with Ovarian Cancer and Benign Ovarian Tumors

There was no significant difference in age, body mass index, menstruation, dysmenorrhea, times of pregnancy, cumulative menstrual years, and marital status between patients with ovarian cancer and benign ovarian tumors (*P* > 0.05). There were significant differences between MRI signs (shape, boundary, enhancement, and tumor components), and ultrasound signs (shape, solid, separated shape, big nipple, and blood supply) in patients with ovarian cancer and benign ovarian tumors (*P* < 0.05). See Table 2.

### 3.3. Multivariate Analysis of Influencing Factors of Ovarian Cancer

Taking ovarian tumors as dependent variables (see Table 3 for assignment) and statistically significant items in Table 2 as independent variables (see Table 3 for assignment), the logistic regression model was used to analyze. The results showed that irregular shape, unclear boundary, obvious enhancement in MRI signs, cystic or solid tumor components, irregular shape, solid features, thick septa, big nipples, and abundant blood supply in ultrasound signs were independent risk factors for ovarian cancer (*P* < 0.05). See Table 4.

### 3.4. Establishment and Analysis of Logistic Regression Model for Diagnosis of Ovarian Cancer

The above risk factors were included in logistic regression analysis, and the regression equation model was established according to the variable regression coefficient table. The regression equation model is as follows: logit (*P*) = −1.153 + [MRI signs : morphology × 1.459 + boundary × 1.549 + reinforcement × 1.492 + tumor components × 1.553] + [ultrasonic signs : morphology × 1.594 + mainly real × 1.417 + separated from × 1.294 + large nipple × 1.271 + blood supply × 1.364]. The logistic regression model for the diagnosis of ovarian cancer was evaluated. The likelihood ratio chi − square = 129.683, DF = 8, and *P* < 0.001, that is, the establishment of the model was statistically significant; Wald chi − square = 138.574, DF = 8, and *P* < 0.001, that is, the coefficient difference of regression equation is statistically significant, suggesting that the construction of logistic regression model is effective. Hosmer lemeshow goodness of fit test shows that the model has good fitting effect, chi − square = 7.539, DF = 7, and *P* = 0.543.

The article "Establishment and Verification of Logistic Regression Model for Qualitative Diagnosis of Ovarian Cancer Based on MRI and Ultrasound Signs" was retracted in 2023. Reasons: signs of a paper mill; compromised peer review; unreliable results or conclusions.

### 3.5. Logistic Regression Model Verification

(1) self-verification: use the logistic regression model to analyze the data and get the diagnostic probability *p* of EA. ROC curve was drawn according to the diagnostic value and true value, and the AUC was 0.883, 95% CI was 0.817 ~ 0.932, diagnostic sensitivity was 93.94%, and specificity was 80.95%, as shown in Figure 1

(2) Out-of-group validation: K-fold cross validation is used to verify the stability of the model. The results show that the training accuracy of 10 groups is 0.904 ± 0.009, and the prediction accuracy is 0.881 ± 0.049, as shown in Table 5.

## 4. Discussion

At present, ovarian cancer has become one of the common tumors that affect women's life quality, and safety [10]. In the deep pelvic cavity, the early stage of the disease lacks typical symptoms and is not easy to detect. When clinical symptoms, such as lower abdominal mass, ascites, and pain appear, the patients with ovarian cancer are already in the middle and late stage of the disease, losing the opportunity of treatment, and the prognosis is not ideal [11]. Therefore, early diagnosis of ovarian cancer is of great value to improve the survival rate and prognosis of patients.

Ultrasound is the preferred imaging examination method for ovarian tumors, which is noninvasive, safe, and simple. It can directly display the internal structure, location, size, shape, and organs involved in the lesions. Combined with color Doppler blood flow imaging technology, we can further understand the distribution of tumor blood vessels and blood flow properties [12, 13]. The results of this study show that the ultrasound manifestations of differentiating malignant tumors from benign tumors are mainly the shape, solid, separated shape, big nipple, and blood supply. Malignant tumors have the ultrasound manifestations of irregular shape, solid, thick separated shape, big nipple, and rich blood supply. Amor et al. [14] put forward six malignant indications of ovarian tumors, namely, septum/wall thickness (≥3 mm), large papillae (≥7 mm), blood flow resistance index < 0.50, central blood flow, solid lesions (cystic part < 50%), and ascites. Abramowicz and Timmerman [15] put forward five malignant signs of ovarian tumors, namely, irregular solid tumors, at least four wall nodules, ascites, maximum diameter ≥ 100 mm, and abundant blood flow signals (blood flow score 4 points). Irregularities in this study include nipple, unsmooth capsule wall, and solid components, which are consistent with the essence of Amor et al. [14]. Some studies have measured the area of solid components (papillae, thick septa, solid tissue, etc.) of ovarian tumors and found that the area of solid tissue is related to the malignant degree of tumors. The larger the area, the larger the solid components and the higher the malignant risk [16]. In this study, solid-solid is an important ultrasonic sign in differentiating benign from malignant tumors, which is consistent with its research. Ultrasound is a classic imaging technique of ovarian tumors, but it has limited function in differentiating benign and malignant tumors due to the influence of low tissue resolution and intestinal gas, and MRI examination is needed when qualitative diagnosis is difficult.

The article "Establishment and Verification of Logistic Regression Model for Qualitative Diagnosis of Ovarian Cancer Based on MRI and Ultrasound Signs" was retracted in 2023. Reasons: signs of a paper mill; compromised peer review; unreliable results or conclusions.

MRI has the characteristics of high soft tissue resolution and multidirectional arbitrary imaging, and with the application of special scanning sequence and dynamic enhancement, it has obvious advantages in locating and characterizing ovarian tumors. The obvious difference of biological characteristics between benign and malignant ovarian tumors is the basis of MRI differential diagnosis [17, 18]. This study shows that irregular shape, unclear boundary, obvious enhancement, cystic, or solid tumor components in MRI signs are independent risk factors of ovarian cancer. Ovarian cancer shows invasive growth, with rapid growth of tumor cells, irregular shape, unclear boundary, and easy invasion of surrounding tissues. At the same time, the blood supply of the tumor is abundant, and it appears obvious enhancement after enhancement [19]. However, benign ovarian tumors show expansive growth, with smooth edges and clear boundaries, mainly cystic components, with thin and regular cyst walls, with little or no enhancement after enhancement [20]. Ovarian cancer is prone to necrosis and hemorrhage. When it is necrotic, it shows uneven low signal intensity on T1WI and high signal intensity on T2WI. When it is bleeding, it shows high signal intensity on T1WI and low signal intensity on T2WI, and both of them have mixed signals [21]. Benign tumors also have signal complexity, such as mucin in mucinous cystadenoma with high signal intensity on T1WI and T2WI, serous cystadenoma with serous components with uniform low signal intensity on T1WI and high signal intensity on T2WI. Mature teratoma contains teeth, sebaceous glands, muscles, etc., showing mixed signals [22]. Therefore, there is a certain risk of misdiagnosis in differentiating benign and malignant ovarian tumors by MRI alone.

The article "Establishment and Verification of Logistic Regression Model for Qualitative Diagnosis of Ovarian Cancer Based on MRI and Ultrasound Signs" was retracted in 2023. Reasons: signs of a paper mill; compromised peer review; unreliable results or conclusions.

This study found that there are significant differences in MRI signs and ultrasound signs in patients with ovarian cancer and benign ovarian tumors. MRI signs include shape, boundary, enhancement, and tumor components. Ultrasound signs include shape, solidity, separation, large nipple, and blood supply. This is consistent with the research results of Cheng Li et al. [22]. They believe that the preoperative use of logistic regression model has a good ability to differentiate between benign and malignant ovarian tumors [22]. Through the results of multivariate logistic regression analysis, this study determined that irregular shape, unclear boundary, obvious enhancement, cystic or solid tumor components in MRI signs and irregular shape, solid dominated, thick septal shape, large nipple, and abundant blood supply in ultrasound signs were independent risk factors for ovarian cancer. Based on this, a regression equation model was established: logit (*P*) = −1.153 + [MRI signs : morphology × 1.459 + boundary × 1.549 + reinforcement × 1.492 + tumor components × 1.553] + [ultrasonic signs : morphology × 1.594 + mainly real × 1.417 + separated form × 1.294 + large nipple × 1.271 + blood supply × 1.364], and the results of self-validation and out-of-group validation of the model show that the model has a good accuracy and stability in the diagnosis of ovarian cancer.

To sum up, irregular shape, unclear boundary, obvious enhancement in MRI signs, cystic or solid tumor components and irregular shape, solid majority, thick septate shape, large nipple, and abundant blood supply in ultrasound signs are independent risk factors for ovarian cancer. After verification, the diagnostic model has good accuracy and stability, which can provide basis for clinical decision-making.

## Figures and Tables

**Figure 1:** ROC curve.

**Table 1:** Clinical baseline data of the patients (*n* = 207).

Index [*n* (%)]	Training group (*n* = 138)	Verification group (*n* = 69)	*t*/*χ*^2^	*P*
Age				
<50 years old	65 (47.10)	35 (50.72)	0.242	0.623
≥50 years old	73 (52.90)	34 (49.28)		
Body mass index				
<23 kg/m^2^	69 (50.00)	32 (46.38)	0.242	0.623
≥23 kg/m^2^	69 (50.00)	37 (53.62)		
Menstruation				
Regular	104 (75.36)	56 (81.16)	0.881	0.348
Irregular	34 (24.64)	13 (18.84)		
Dysmenorrhea				
Not have	125 (90.58)	61 (88.41)	0.239	0.625
Have	13 (9.42)	8 (11.59)		
Number of pregnancies				
<2	64 (46.38)	36 (52.17)	0.619	0.431
≥ 2	74 (53.62)	33 (47.83)		
Cumulative menstrual years				
<30	55 (39.86)	30 (43.48)	0.250	0.617
≥30	83 (60.14)	39 (56.52)		
Marital status				
Unmarried	13 (9.42)	7 (10.14)	1.095	0.578
Married	121 (87.68)	58 (84.06)		
Other	4 (2.90)	4 (5.80)		
Tumor nature				
Ovarian cancer	33 (23.91)	18 (26.09)	0.117	0.732
Benign ovarian tumor	105 (76.09)	51 (73.91)		

The article "Establishment and Verification of Logistic Regression Model for Qualitative Diagnosis of Ovarian Cancer Based on MRI and Ultrasound Signs" was retracted in 2023. Reasons: signs of a paper mill; compromised peer review; unreliable results or conclusions.

**Table 2:** Clinical data of patients with ovarian cancer and benign ovarian tumors(*n* = 138).

Index [*n* (%)]	Ovarian cancer (*n* = 33)	Benign ovarian tumor (*n* = 105)	*t*/*χ*^2^	*P*
Age				
<50years old	16 (48.48)	49 (46.67)	0.033	0.855
≥50years old	17 (51.52)	56 (53.33)		
Body mass index				
<23 kg/m^2^	18 (54.55)	51 (48.57)	0.358	0.549
≥23 kg/m^2^	15 (45.45)	54 (51.43)		
Menstruation				
Regular	23 (69.70)	81 (77.14)	0.750	0.387
Irregular	10 (30.30)	24 (22.86)		
Dysmenorrhea				
Not have	29 (87.88)	96 (91.43)	0.072	0.789
Have	4 (12.12)	9 (8.57)		
Number of pregnancies				
<2	14 (42.42)	50 (47.62)	0.273	0.602
≥ 2	19 (57.58)	55 (52.38)		
Cumulative menstrual years				
<30	13 (39.39)	42 (40.00)	0.004	0.951
≥30	20 (60.61)	63 (60.00)		
Marital status				
Unmarried	3 (9.09)	10 (9.52)	0.008	0.996
Married	29 (87.88)	92 (87.62)		
Other	1 (3.03)	3 (2.86)		
Ultrasonic signs				
Regular	16 (48.48)	77 (73.33)	7.055	0.008
Irregular	17 (51.52)	28 (26.67)		
Real-oriented				
Yes	19 (57.58)	4 (3.81)	52.261	<0.001
No	14 (42.42)	101 (96.19)		
Separation form				
Thick	26 (78.79)	12 (11.43)	57.095	<0.001
None or thin	7 (21.21)	93 (88.57)		
Big nipple				
Yes	16 (48.48)	12 (11.43)	21.318	<0.001
No	17 (51.52)	93 (88.57)		
Blood supply				
Little or no	1 (3.03)	22 (20.95)	5.807	0.016
Enrich	32 (96.97)	83 (79.05)		
MRI signs				
Regular	8 (24.24)	99 (94.29)	70.725	<0.001
Irregular	25 (75.76)	6 (5.71)		
Boundary				
Clear	10 (30.30)	105 (100.00)	87.818	<0.001
Unclear	23 (69.70)	0 (0.00)		
Strengthen				
Obvious	33 (100.00)	19 (18.10)	71.730	<0.001
Mild or none	0 (0.00)	86 (81.90)		
Tumor component				
Cystic	0 (0.00)	92 (84.62)	86.743	<0.001
Capsule or substantiality	33 (100.00)	13 (12.38)		
T_1_WI				
Low signal	19 (57.58)	39 (37.14)	4.425	0.109
High signal	1 (3.03)	7 (6.67)		
Hybrid signal	13 (39.39)	59 (56.19)		
T_2_WI				
High signal	25 (75.76)	61 (58.10)	3.336	0.068
Hybrid signal	8 (24.24)	44 (41.90)		

The article "Establishment and Verification of Logistic Regression Model for Qualitative Diagnosis of Ovarian Cancer Based on MRI and Ultrasound Signs" was retracted in 2023. Reasons: signs of a paper mill; compromised peer review; unreliable results or conclusions.

**Table 3:** Assignment.

Variable	Assignment
Dependent variable	Benign ovarian tumor = 1, ovarian cancer = 2
Independent variable	
MRI signs	
Form	Regular = 1, irregular = 2
Boundary	Clear = 1, unclear = 2
Strengthen	Mild or none = 0, obvious = 1
Tumor component	Cystic = 1, capsule or substantiality = 2
Ultrasonic signs	
Form	Regular = 1, irregular = 2
Real-oriented	No = 0, yes = 1
Separation form	None or thin = 0, thick = 1
Big nipple	No = 0, yes = 1
Blood supply	Little or no = 0, enrich = 1

**Table 4:** Multivariate analysis of influencing factors of ovarian cancer (*n* = 138).

Factors	*β*	S. E.	*Waldχ* ^2^	*P*	OR	95% CI
MRI signs						
Form	1.459	0.475	9.435	<0.001	4.302	2.594 ~ 7.136
Boundary	1.549	0.513	9.117	<0.001	4.707	3.058 ~ 7.251
Strengthen	1.492	0.655	5.189	0.002	4.446	2.836 ~ 6.972
Tumor component	1.553	0.538	8.333	<0.001	4.726	3.147 ~ 7.096
Ultrasonic signs						
Form	1.594	0.487	10.713	<0.001	4.923	3.529 ~ 6.863
Real-oriented	1.417	0.471	9.051	<0.001	4.125	2.463 ~ 6.912
Separation form	1.294	0.593	4.762	0.010	3.647	1.894 ~ 7.025
Big nipple	1.271	0.581	4.786	0.009	3.564	2.029 ~ 6.265
Blood supply	1.364	0.465	8.604	<0.001	3.912	2.351 ~ 6.514

**Table 5:** K-fold cross validation (*n* = 69).

Group number	Prediction accuracy	Training accuracy
1	0.921	0.930
2	0.950	0.938
3	0.913	0.920
4	0.894	0.905
5	0.851	0.882
6	0.926	0.937
7	0.908	0.925
8	0.883	0.914
9	0.852	0.865
10	0.847	0.891
$\;\bar{x}\pm \text{s}$	0.881 ± 0.049	0.904 ± 0.009

## Data Availability

The labeled dataset used to support the findings of this study is available from the corresponding author upon request.
